The article "Design and Experiment of Assistive Mechanism for Adjustment of Transrectal Ultrasound Probe" was published in 2020. Journal: Appl Bionics Biomech.

# Design and Experiment of Assistive Mechanism for Adjustment of Transrectal Ultrasound Probe

**DOI:** 10.1155/2020/8846073

**Published:** 2020-10-15

**Authors:** Jin-Gang Jiang, Hui Zuo, Yong-De Zhang, Zhi-Yuan Huang, Xiao-Wei Guo, Yong Xu

**Affiliations:** ^1^Key Laboratory of Advanced Manufacturing and Intelligent Technology, Ministry of Education, Harbin University of Science and Technology, Harbin 150080, China; ^2^Robotics & its Engineering Research Center, Harbin University of Science and Technology, Harbin 150080, China; ^3^Urinary Surgery, The General Hospital of Chinese People's Liberation Army, Beijing 100039, China

## Abstract

Transrectal ultrasound prostate biopsy is the most commonly used method for the diagnosis of prostate cancer. During the operation, the doctor needs to manually adjust the ultrasound probe for repeated adjustments, which is difficult to ensure the efficiency, accuracy, and safety of the operation. This paper presents a passive posture adjusting mechanism of transrectal ultrasound probe. The overall mechanism has 7 degrees of freedom, consisting of a position adjustment module, a posture adjustment module, and an ultrasonic probe rotation and feed module. In order to achieve the centering function, the posture adjustment module is designed based on the double parallelogram. Centering performance is verified based on SimMechanics, and remote center point error of physical prototypes is evaluated. The maximum error of the azimuth remote center point motion and the maximum error of the remote center point motion of the ultrasonic probe are 4 mm and 3.4 mm, respectively, which are less than the anus that can withstand 6 mm. Meanwhile, the analysis of measurement error shows that the random error correlation is weak in different directions, the systematic error confidence intervals of azimuth and elevation angle are less than 2.5 mm, and the maximum relative fixed point error and the maximum relative standard error are 14.73% and 14.98%, respectively. The simulation and testing results have shown the effectiveness and reliability of the propose mechanism.

## 1. Introduction

Nowadays, people are paying attention to their own health problems as the significant improvement in people's living standards. The American Cancer Society counts the top ten cancers with the highest cancer incidence in the United States in 2017. Prostate cancer ranks first among all high-risk cancers among men, accounting for about one-fifth of the total number of male cancer patients; thus, it will cause great pain to male patients. At the same time, the mortality rate of prostate cancer is increasing at a rate of 2% per year and showing a trend of rejuvenation [1, 2]. The most critical means of curing prostate cancer is early diagnosis [3–8].

In the clinic, the most common method for early diagnosis of prostate cancer is transrectal ultrasound prostate biopsy. An ultrasound probe is utilized to probe the patient's rectum and puncture the prostate under ultrasound-guided guidance when the operation is performed. However, this surgery still has the following problems: the entire procedure requires the doctor to operate with an ultrasound probe, and it is necessary to repeatedly adjust the ultrasound probe, which may cause fatigue and mood swings; the ultrasound probe needs to be inserted into the patient's rectum, which will cause damage to the anus when adjusting the posture of the probe; this surgical procedure requires the cooperation of multiple nurses, resulting in wastage of personnel. Moreover, the number of prostate patients is growing, and the existing medical staff is not enough to complete such a large workload, and the traditional hand-held method is difficult to ensure the precision of the puncture intervention because of the special location of the prostate. Therefore, it is necessary to study medical devices that assist doctors in prostate scans and biopsy gun puncture interventions.

In recent years, minimally invasive interventional robotics has gradually become one of the hotspots in the medical field, and this technology has attracted the attention of researchers. In 2007, Yan Yu of Thomas Jefferson University in the United States developed a prostate seed implantation treatment system based on ultrasound image navigation [9–11], which can automatically or manually use the rotation operation to obtain ultrasound images of lesion points. The American Engineering Research Center and Johns Hopkins University have jointly developed a robotic system that includes ultrasound image navigation and TPS to enable free movement and attitude adjustment of the biopsy needle in a vertical plane [12, 13]. An ultrasound imaging-guided prostate interventional robot was designed by Kim et al., in which 2-DOF is able to be manually adjusted for posture adjustment, and two degrees of freedom are used to adjust the movement and rotation of the ultrasound probe [14]. Vitrani et al. of the University of Pittsburgh designed an artificially operated prostate biopsy probe holder, and its structural is similar to a 6-DOF series manipulator, which uses ultrasound transrectal puncture for good stiffness and stability [15]. The Institute of Intelligent Machines of Harbin University of Science and Technology has designed the structure of an all-round prostate robot. This error of each axis of the system is kept within 0.05 mm through experiments, which has high repeat positioning accuracy and meet the surgical requirements [16–18].

At present, the active prostate interventional robot has been extensively studied; however, it is difficult to promote and apply because of its complicated system, high cost, and long training time [19]. In contrast, passive prostate-assisted interventional mechanism has relatively simple structure, a short design cycle, low cost, and is easier to promote and apply than active mechanism.

The key technology of the passive prostate-assisted interventional mechanism is the centering motion of the transrectal ultrasound probe, and the remote center mechanism (RCM) can realize the centering motion of the ultrasound probe, so that the doctor's hands are truly liberated. The concept of the RCM was first proposed by Taylor et al. at Johns Hopkins University in 1995. The designed azimuth rotation center and the pitch angle rotation center intersect at the remote center point, and the posture of the puncture needle can be arbitrarily adjusted in 2-DOF, and the purpose of adjusting the distal center position is achieved by the expansion and contraction of the link [20]. The American Computer Surgery Systems Research Center and Johns Hopkins University have developed a renal puncture robot that is able to be installed on a surgical bed. In this robot, a single-bar parallelogram RCM mechanism is used to complete the centering rotation function during the operation [21]. Jilin University developed a mirror arm of a new type of surgical robot based on RCM. This RCM uses the crank slider to realize the centering function of the actuator [22]. Kuo and Dai designed a decoupling RCM based on a parallel arm. The mechanism includes a fixed base, a motion restraining leg, and two auxiliary drive legs. The motion-constrained leg is designed as a 3RP mechanism, which can realize the rotational motion and axial translational motion of the surgical instrument about the rotation axis [23].

From the research status, it can be found that the existing RCM can meet the surgical requirements. However, the lack of work concerning on a single-bar parallelogram mechanism, a crank slider mechanism, or a triangular mechanism is partly due to complicated structure, poor stability, and large space occupation.

This paper is aimed at studying the ultrasonic probe position and posture adjustment mechanism with centering function and passive. The range of motion of the ultrasonic probe, the operable space of the mechanism, and the design criteria were obtained accordingly to analyze the surgical procedure of prostate biopsy. The mechanism is divided into functions, and the degree of freedom of each module is allocated reasonably according to the design criteria. Next, each module of the mechanism is designed and, a three-dimensional model of the overall mechanism is drawn. This study is focused on designing the posture adjustment module with centering function in design phase. The D-H method is utilized to establish the coordinate system of the mechanism, and the joint parameters are obtained. Combined with the simulation results, the positioning error of the remote center point and the analysis of error in the actual surgical operation were tested and analyzed in the experimental part.

The transrectal ultrasound probe position-adjusting RCM will complement a large gap in the passive prostate-assisted interventional mechanism in the field of prostate intervention. The designed RCM can not only enable doctors to truly liberate their hands during the operation, but also achieve the level of planning and industrialization, improve the efficiency and precision of prostate interventional surgery, and a more practical motivation for this study is to promote the development of prostate cancer medicine.

## 2. Methods

### 2.1. Analysis of Functional Requirements of Adjustment Mechanism

Transrectal prostate biopsy is an effective means of diagnosing prostate cancer. When the operation is performed, the doctor uses an ultrasound probe to probe the patient's rectum and puncture the prostate under the guidance of ultrasound images.

#### 2.1.1. Motion Analysis of Ultrasonic Probe

The prostate, which closes to the rectal wall, is located in the abdomen of the rectum. The upper end of the prostatic body has a transverse diameter of about 40 mm, a vertical diameter of about 30 mm, and anteroposterior diameter of about 25 mm. After filling with water, the volume increases by 25%. The cavity rectal ultrasound probe is invaded through the anus. During the guided puncture, the rectal ultrasound probe needs to perform position adjustment, azimuth adjustment, pitch adjustment, rotation, and feed to achieve multiangle omnidirectional scanning of the prostate. The rectal anatomy is shown in Figure 1. We found that the ampulla space inside the rectum is relatively wide; however, the anal internal sphincter is muscle and its space is narrow, and the position is fixed.

The ultrasound probe pass through the anal canal to reach the ampulla of the rectum, and the ultrasound probe contacts with the internal sphincter of the anus at the anal canal. Therefore, the ultrasound probe should always swing with the center of the anus peripheral as the center of rotation to avoid damage to the rectum and increase the patient's pain when scanning the prostate.  Figure 2 shows that the resulting range of motion is a conical space.

#### 2.1.2. Analysis of Mechanism Operational Space

During the prostate biopsy operation, the patient adopts the left lateral position. In order to prevent the ultrasound probe from interfering with the bed during adjustment, the patient keeps knee-shouldered and the buttocks are positioned the bedside. The posture of the patient is shown in Figure 3. The longitudinal axis of the trunk is 30°~45° to the edge of the bed, the angle between the thigh and the edge of the bed is 45°~60°, and the distance between the prostate and the bed is 150~250 mm. The anus is able to be exposed according to the position of left knee flexing. Furthermore, it is convenient for the ultrasound probe to be invaded from the rectum.

#### 2.1.3. Design Guidelines of Position and Posture Adjustment Mechanism

According to the surgical characteristics of transrectal ultrasound probe prostate biopsy surgery, the design of the ultrasonic probe posture adjustment mechanism needs to be considered as following below criteria:

1. *Continuous Motion*: The mechanism should continuously move, which can drive the ultrasonic probe to smoothly reach the required spatial position and posture
2. *Reliable Locking*: In order to the safety and positioning accuracy of the operation, the mechanism needs to be securely locked when the ultrasonic probe moves to a proper posture
3. The positioning mechanism and the posture adjustment mechanism are not interfere with each other and are completely decoupled
4. The working range is able to cover all prostate areas without blind spots
5. The structure is simple and reliable, and the manufacturing is easy obtained

### 2.2. Design of Position and Posture of Adjustment Mechanism

In order to meet the needs of different scanning range of prostate tissue by ultrasound probe during operation, the position adjustment function, posture adjustment function, rotation, and feed function of the ultrasonic probe should be realized. The 3-DOF spatial positioning mechanism, 2-DOF posture adjustment mechanism, and 2-DOF ultrasonic probe rotation and feed mechanism are adopted. The motion relationship between the three mechanisms is completely decoupled. The transrectal ultrasound probe position and posture adjustment mechanism are composed of a position adjustment module, a posture adjustment module, an ultrasonic probe rotation, and a feed module and a bottom clamping device. From the perspective of degree of freedom, this adjustment mechanism is a 7-DOF robot. Joint 7 is only a moving joint, and the other joints are rotating joints in the mechanism. The joints 1 to 4 constitute a position adjustment module; joint 5 and joint 6 constitute a posture adjustment module; joint 7 is utilized to realize the penetration movement of the ultrasonic probe along the peripheral center of the anus, and the joint 8 is utilized to realize the rotation of the ultrasonic probe around its own axis.  Figure 4 shows schematic diagram of each module of the adjustment mechanism.

The centering function is implemented by the posture adjustment module. We need to consider the centering effect and the implementation of the centering function; therefore, the design of posture adjustment module is focused in design phase.

Due to the size and weight of the posture adjustment module affect the size of the position adjustment module, the specific structural size of the posture adjustment module is calculated in this section. For the posture adjustment module, the 2-DOF structure is chosen. In order to make the ultrasound probe move in two directions around the center of the anus, an RCM mechanism is considered. The posture adjustment module adopts an RCM mechanism based on double parallelograms, and its schematic diagram is shown in Figure 5. Double parallelograms are ▱ADCF and ▱BCIJ. In order to conveniently describe the characteristics of the mechanism, a local coordinate system is established in Figure 5. When the link DF swings the angle *α* around the point D, the double parallelogram mechanism has the following characteristics:

1. *Parallel Characteristics*: *AD*//*BI*//*CJ* and *AC*//*DF*//*IJ*
2. *Centering Characteristics*: The position of the intersection *H* of the *AD* extension line and the *JI* extension line is always unchanged

When the doctor performs the operation, the fixed point *H* is always at the center point of the anus, and the *AD* rod is vertically above the patient's ankle. The length *DH* must be greater than half the width of the patient's ankle to prevent the posture adjustment module from interfering with the patient's body. According to the size of the human body, the width of the crotch is generally 300 mm~420 mm, so the length of *DH* needs to satisfy the equation:

(1) $$\begin{array}{c} l_{DH}>210\text{mm}. \end{array}$$

We choose*l*_*DH*_ = 220mm and *l*_*AD*_ = 30mm, and then, the length of the longitudinal link is as follows:

(2) $$\begin{array}{c} l_{BI}=250\text{mm}. \end{array}$$

The size of the vertical plane of the anus peripheral center point is 120 mm away from the buttocks. In order to prevent the longitudinal link *BI* from interfering with the patient's body, the length *HI* needs to satisfy the equation:

(3) $$\begin{array}{c} l_{HI}>120\text{mm} \end{array}$$

Taking into account the ultrasonic probe rotation and the size occupied by the feed module, we choose *l*_*DI*_ = 200mm, *l*_*IJ*_ = 30mm, the length of the transverse link is:

(4) $$\begin{array}{c} l_{AC}=230\text{mm} \end{array}$$

According to the physiological characteristics of the human body, the space occupied by the prostate is generally 40 mm × 30 mm × 25 mm, and Figure 6 shows the spatial state of the prostate in the left lateral position and the spatial analysis of the angle of the ultrasound probe scanning the prostate. The azimuth angle *β* is the swing angle of the ultrasonic probe in the transverse section, and the pitch angle *γ* is the swing angle of the ultrasonic probe in the longitudinal section. Due to the distance *HK* from the peripheral center point *H* of the anus to the surface of the prostate is 60 mm, the volume of the prostate is increased by 25% after filling with water, and the volume of the prostate is 50 mm × 40 mm × 40 mm when calculating the swing angle of the ultrasonic probe.

Therefore, *PK* = 25mm, *MK* = *NK* = 40mm, $OM=OK=1/2MN=1/2\sqrt{{MK}^{2}+{NK}^{2}}=28\text{mm}$,

(5) $$\begin{array}{c} OH=HK+OK=88\text{mm}. \end{array}$$

In order for the ultrasound probe to cover the entire area of the prostate, the beta and gamma angles should satisfy the following equation:

(6) $$\begin{array}{c} \tan\frac{\beta }{2}\geq \frac{OM}{OH}=\frac{28}{88},\\ \tan\frac{\gamma }{2}\geq \frac{PK}{HK}=\frac{25}{60}. \end{array}$$

Solving result is *β* ≥ 35.4°, *γ* ≥ 45.3°.

### 2.3. Simulation Analysis of the Motion Performance of Adjustment Mechanism

The principle design of the ultrasonic probe position and posture adjustment mechanism determines the overall configuration of the mechanism, so that the designed mechanism is able to meet the working requirements, which meet the scanning range of the ultrasound probe during the operation to completely cover every part of the prostate. Therefore, it is necessary to utilize kinematics to analyze the mechanism to solve the motion space of the mechanism and the centering effect when the ultrasonic probe finishes the adjustment of posture.

#### 2.3.1. Coordinate System Establishment and Joint Parameters

According to the structure of the ultrasonic probe position and posture adjustment mechanism, a schematic diagram of the mechanism is established, as shown in Figure 7. This mechanism is a six-bar linkage consisting of two parallelograms because of the posture adjustment module is not a simple open-loop kinematic chain.

In this mechanism, the rod 6 and the rod 7 are, respectively, the probe rotation and feed module mounting platform and the feeding platform, and the rod 8 is an ultrasonic probe. The coordinate system origin *o*_6_ of the rod 6 is established at the remote center point based on the analysis of the mechanism characteristics. The coordinate system origin *o*_7_ of the rod 7 is established at the end of the feed platform, and the coordinate system origin *o*_8_ of the rod 8 is established at the end of the ultrasonic probe, and the directions of the *x*_6_-axis and the *x*_7_-axis are along the ultrasonic probe axis *x*_8_. Therefore, the system is regarded as a simple open-loop kinematic chain to discuss and research; furthermore, the D-H method is utilized to solve the kinematics of the mechanism.

The base coordinate system is *o*_0_*x*_0_*y*_0_*z*_0_, and *d*_1_, *a*_1_, *a*_2_, *a*_3_, *a*_4_, *a*_6_, and *a*_7_ are the rod lengths of the respective links, and *θ*_1_, *θ*_2_, *θ*_3_, and *θ*_4_ are the rotation angles of the respective rotary joints of the position adjustment mechanism, respectively.

Due to the rod 2 that constitutes a parallelogram structure, *θ*_3_ = −*θ*_2_, *θ*_5_, *θ*_6_ are the azimuth and pitching angles of the RCM mechanism, *a*_7_ is the feed distance of the ultrasonic probe along the *x*_8_-axis, and *α*_7_ is the rotation angle of the ultrasonic probe. According to the designed requirements, the organization has a total of 7 degrees of freedom, and the joint parameters are shown in Table 1.

#### 2.3.2. Simulation of Centering Effect Based on SimMechanics

According to the mechanism diagram and the connecting rod parameters drawn in Figure 7 and Table 1, the physical model of the ultrasonic probe posture adjustment mechanism is established in the SimMechanics toolbox, the end track of the ultrasonic probe is tracked, and we output the recorded position coordinates to Workspace for drawing 3D graphics.

The model established for the ultrasonic probe pose adjustment mechanism in the SimMechanics toolbox is shown in Figure 8. The SimMechanics model mainly includes a ground module, 13 rigid body modules, 12 rotary joint modules, 1 moving joint module, 6 drive modules, and 2 sensor modules.

1. “World” indicates the position of the base coordinate system, which is located on the bottom surface of the column
2. The rigid body modules respectively represent 13 movable members of the posture adjustment mechanism
3. The rotary joints respectively represent the movement relationship between the members as rotation
4. The moving joints represent the rotation and advancement of the ultrasonic probe
5. The movement constraint of the module relative to the posture adjustment module is provided
6. The drive modules are respectively added to the corresponding joints
7. The sensor modules respectively record the coordinate positions that the end position of the ultrasonic probe and the position of reached handheld

The posture adjustment module enables the ultrasonic probe to realize the centering function of swinging around a certain point and simulates the centering effect of the ultrasonic probe.  Table 2 shows the setting parameters.

## 3. Results

### 3.1. Simulation Results of Centering Effect

The simulation results when the feed distance *a*_6_ = 0 mm are shown in Figure 9. The posture adjustment module allows the ultrasonic probe to realize the centering function of swinging around a certain point, and the effectiveness of centering the ultrasonic probe is simulated. The parameter settings are shown in Table 2.

The simulation results when the feed distance *a*_6_ = 0 mm are shown in Figure 9. The color line segments in the figure represent the posture of the ultrasonic probe at different joint angles. The position coordinates of the remote center point of the mechanism are (381.000, 2.461, and 210.800) when *θ*_1_ = −30°, *θ*_2_ = 20°, and *θ*_4_ = 80°. The scanning end of the ultrasonic probe is always at the remote center point of the mechanism, and a cone-shaped space with the point as a vertex is formed when the azimuth and pitching angles are adjusted according to a given angle.

The omnidirectional scan of the prostate can be completed when the doctor inserts the ultrasound probe into the rectum and adjusts the azimuth, pitching angle, and the angle of rotation of the ultrasound probe. The joint parameters of the position adjustment module and the posture adjustment module are not changed in order to observe the change in the posture after the ultrasonic probe is fed. The feed distance of the ultrasonic probe was changed to *a*_6_ = 30 mm. The simulation results obtained are shown in Figure 10.

Measurements showed that the coordinates of this point remained at (381.000, 2.461, and 210.800). The ultrasonic probe still changed the azimuth and pitching angles according to the remote center point after feeding 30 mm, which meets the design requirements. We changed the feed distance of the ultrasonic probe to *a*_6_ = 60 mm, while leaving the parameters of the other joints unchanged, and the posture change of the ultrasonic probe was simulated. The simulation results are shown in Figure 11. It can be seen in the figure that the coordinates of the intersections of all the line segments intersecting in space remain at (381.000, 2.461, and 210.800). This means that the azimuth and pitching angles of the ultrasonic probe remain changed according to the remote center point after feeding 60 mm, which also meets the design requirements.

The results of the simulation of the ultrasonic probe at feed rates of 0 mm, 30 mm, and 60 mm, respectively, showed that the ultrasonic probe can achieve a very stable centering effect at different feed rates and can be used for surgery.

### 3.2. Experiment Results of Centering Effect

#### 3.2.1. Physical Prototype of the Posture Adjustment Mechanism of Ultrasonic Probe

Many interference factors exist because the mechanism is operated during the actual operation. This experimental section describes the simulation of the actual surgical environment and operation process. The range and continuity of each joint, reliable locking ability, position adjustment mechanism working space and positioning ability, mechanism static stiffness, RCM posture adjustment, and centering motion performance were tested to verify the rationality of these mechanisms.  Figure 12 shows the physical prototype of the mechanism.

#### 3.2.2. Remote Center Point Error Measurement

The doctor adjusts the azimuth and pitching angle of the ultrasound probe to omnidirectionally scan the prostate. To ensure the safety of the operation and reduce the damage caused to the patient by the ultrasonic probe, the ultrasonic probe needs to achieve a centering motion around the center of the anus. Therefore, it was necessary to test the RCM of the posture adjustment module to examine whether it meets the surgical requirements.

The RCM performance comprises the displacement range of the remote center point of the mechanism in the space when the ultrasonic probe performs posture adjustment. The RCM performance can be evaluated by measuring the error between the spatial fixed point and the remote center marked point under the existing experimental conditions. A fixed point in space measures only the error of the remote center point in the two-dimensional (2D) plane because the position change of the remote center point is 3D in space. Therefore, in this section, we describe two sets of experiments performed to measure the error, which is caused by changing the azimuth or pitching angle, separately.

*(1) Azimuth Remote Center Point Motion Error Measurement*. The azimuth angles *θ*_5_ (-40°, -20°, 0°, 20°, and 40°) were adjusted under different feed rates *a*_6_ (0 mm, 30 mm, and 60 mm). The mechanism was adjusted to a certain position, and then, the joints of the position adjustment mechanism were locked. The pitch angle of the ultrasonic probe was *θ*_6_ = 0°, and the rotation angle of the ultrasonic probe *α*_7_ = 0°. Because the azimuth is adjusted to the angle change in the horizontal plane, the wooden board with the coordinate paper was fixed directly below the ultrasonic probe (the scale of the coordinate paper was 1 mm), and then, the position of the remote center point was marked on the ultrasonic probe; a laser was used to illuminate the remote center point as a fixed spatial point. Finally, the position of the fixed spatial point was marked on the coordinate paper.  Figure 13 shows experimental process.

The experimental data were obtained by means of multiple measurements. The experimental results are shown in Figure 14. The points marked on the coordinate paper were enlarged and measured. The distance between the subsequent remote center point and the fixed spatial point is less than 4 mm, and the deformation of the anus is about 6 mm. Therefore, the accuracy of the remote center point under the azimuth angle meets the surgical requirements.

*(2) Pitch Angle Remote Center Point Motion Error Measurement*. The pitch angles *θ*_6_ (-24°, -12°, 0°, 12°, and 24°) were adjusted under different feed rates *a*_6_ (0 mm, 30 mm, and 60 mm). The mechanism was adjusted to a certain position, and then, the joints of the position adjustment mechanism were locked. The pitch angle of the ultrasonic probe was *θ*_5_ = 0°, and the rotation angle of the ultrasonic probe *α*_7_ = 0°. Because the azimuth is adjusted to the angle change in the vertical plane, the wooden board with the coordinate paper was fixed directly below the ultrasonic probe (the scale of the coordinate paper was 1 mm), and then, the position of the remote center point was marked on the ultrasonic probe; a laser was used to illuminate the remote center point as a fixed spatial point. Finally, the position of the fixed spatial point was marked on the coordinate paper.  Figure 15 shows the experimental process. The obtained experimental data are shown in Figure 16.

The measurement of the points marked on the coordinate paper showed that the distance between the subsequent remote center points and the fixed spatial point is less than 3.4 mm, and the deformation of the anus is about 6 mm. Therefore, the accuracy of the remote center point meets the surgical requirements under the change in the pitch angle.

## 4. Discussion

The positioning error of the remote center point is related to the entire mechanism and is composed mainly of systematic error and random error.

The systematic error is composed of multiple error factors with deterministic changes [24–26]. Therefore, we used the measured mean and variance to consider the systematic error, and, in order to avoid the error estimation bias caused by the small number of sample repetitions, the confidence interval was used to state the systematic error limit. Then, we defined the safety factor as*k*_1_ and $\left[\bar{x}-k_{1}s,\bar{x}+k_{1}s\right]$ as the confidence interval for*μ*, where*μ*is the mean, *s* is the measurement variance, and$\bar{x}$is the unbiased estimator of*μ*. In addition, in order to determine the relative error, the relative fixed point error and the relative standard deviation (RSD) were used as the evaluation indexes in each direction. The relative fixed point error*ε*_0_is the error of the measured mean value with respect to the fixed point. It takes the relative error of the *x*-axis coordinates as an example, which is expressed as

(7) $$\begin{array}{c} \varepsilon_{0}=\frac{\left|\bar{x}-x_{0}\right|}{x_{0}}\times 100\%, \end{array}$$

where $\bar{x}=\sum_{i=1}^{n}x_{i}/n$, and*x*_0_is the *x*-axis coordinate value of the fixed point.

The RSD can be used to verify the precision of the measurement results:

(8) $$\begin{array}{c} \text{RSD}=\frac{S}{\bar{x}}\times 100\%. \end{array}$$

Most random errors follow a normal distribution. To reflect the spatial relationship of random stochastic processes in different spatial locations, the value of the random error parameters ranged from -1 to 1 [27, 28]. The *x* and *y* direction and the *x* and *z* directions of the azimuth and pitching angles were used as the positioning quality indicators as two sets of 2D random variables. The correlation coefficient between 2D variables is defined as

(9) $$\begin{array}{c} r=\frac{\sum_{i=1}^{n}\left(x_{i}-\bar{x}\right)\left(y_{i}-\bar{y}\right)}{\sqrt{\sum_{i=1}^{n}{\left(x_{i}-\bar{x}\right)}^{2}\sum_{i=1}^{n}{\left(y_{i}-\bar{y}\right)}^{2}}}. \end{array}$$

According to the theory of the above error analysis, the confidence interval was taken as 90%, and the measured mean value, relative fixed point error, relative standard error, confidence interval, and 2D variable relative parameters were calculated. The azimuth error calculation results are shown in Table 3.

As shown in Table 3, for the same probe feed distance, the width of the confidence interval between the *x* direction and the *y* direction is close, and both are stable at approximately 2.3 mm, indicating that the positioning performance is relatively stable. The relative fixed point error and RSD in different feed directions are basically stable in the *x* direction, and the relative fixed point error is larger in the *y* direction, except in the case of the 0 mm feed distance. However, for the remaining feed distances, the error remains stable below 15%, and the error can be controlled within 1.8 mm. The relative error parameters of the *x* and *y* directions under different feed distances are relatively low, indicating that the correlation between the two parameters is not strong. It is proved that the measurement value in the *y* direction cannot be determined by measuring the *x* direction. The results show that the azimuth centering performance is stable, and the accuracy meets the requirements. Similarly, an error analysis of the remote center point measurement data was performed. The analysis results are shown in Table 4.

## 5. Conclusions

This study is aimed at designing a passive ultrasound probe position and posture adjustment mechanism to assist doctors performing prostate scans and puncture interventions. In this paper, the forward kinematics analysis of the mechanism, the simulation of the centering effect, the development of the physical prototype, and related experimental research were presented. The main findings are as follows.

1. The moving shape of the ultrasonic probe is the conical space around the center of rotation of the anus. The design requirements are determined by analyzing the surgical procedure; the posture adjustment module is designed such that the double parallel quadrilateral RCM mechanism allows the ultrasonic probe to achieve the centering function
2. SimMechanics was used to simulate the effectiveness of centering the ultrasonic probe when adjusting the posture under different feed distances. The study results showed that the ultrasonic probe is centered and stable, which verifies that the position adjustment of the ultrasonic probe meets the design requirements
3. A physical prototype was developed and debugged. The effectiveness of the centering of the remote center point was measured when adjusting the posture of the ultrasonic probe, and the displacement range of the remote center point in space was obtained. The experimental results show that the maximum error of the azimuth remote center point motion and the maximum error of the remote center point motion of the ultrasonic probe are 4 mm and 3.4 mm, respectively, that is, less than a 6 mm anus can withstand. The random error correlation in different directions is weak, the systematic error confidence intervals of the azimuth and elevation angle are less than 2.5 mm, and the maximum relative fixed point error and the maximum relative standard error are 14.73% and 14.98%, respectively

The system meets the surgical requirements of a passive medical mechanism to be applied in actual surgical procedures.

## Figures and Tables

**Figure 1:** Rectum anatomy graph.

**Figure 2:** Motion scope of ultrasonic probe.

**Figure 3:** Operational space.

**Figure 4:** Schematic diagram of the position adjustment mechanism of the transrectal ultrasound probe and each module structure diagram.

**Figure 5:** Schematic diagram of posture adjustment module.

**Figure 6:** Analysis of swing angle of ultrasonic probe.

**Figure 7:** The kinematics coordinate system.

**Figure 8:** SimMechanics model of ultrasonic probe position adjustment mechanism.

**Figure 9:** Posture of ultrasonic probe at 0 mm feeding: (a) three-dimensional map; (b) *xoy* plane projection; (c) *yoz* plane projection; and (d) *xoz* plane projection.

**Figure 10:** Posture of ultrasonic probe at 30 mm feeding: (a) three-dimensional map; (b) *xoy* plane projection; (c) *yoz* plane projection; and (d) *xoz* plane projection.

**Figure 11:** Posture of ultrasonic probe at 60 mm feeding: (a) three-dimensional map; (b) *xoy* plane projection; (c) *yoz* plane projection; and (d) *xoz* plane projection.

**Figure 12:** Physical prototype of the posture adjustment mechanism of ultrasonic probe.

**Figure 13:** Measurement of azimuth remote center point error: (a) overall view; (b) partial magnification view.

**Figure 14:** Remote center point error under the motion of azimuth angle.

**Figure 15:** Measurement of pitching center point error: (a) overall view; (b) partial magnification view.

**Figure 16:** Remote center point error under the motion of pitching angle.

**Table 1:** D-H parameters of manipulator.

Rod *i*	1	2	3	4	5	6	7	8
*a*_*i*−1_ (°)	0	29.5	200	29.5	250	300	*a*_6_	190
*α*_*i*−1_ (°)	0	-90	0	90	0	90	0	*α*_7_
*d*_*i*_ (mm)	445	0	0	0	0	0	0	0
*θ*_*i*_ (°)	*θ*_1_	*θ*_2_	−*θ*_2_	*θ*_4_	*θ*_5_	*θ*_6_	0	0

**Table 2:** Posture simulation parameters of ultrasonic probe at 0 mm, 30 mm, and 60 mm feeding.

*θ*_1_ (°)	*θ*_2_ (°)	*θ*_4_ (°)	*θ*_5_ (°)	*θ*_6_ (°)	*α*_7_ (°)
-30	20	80	-20~20	-25~25	0

**Table 3:** Analysis result of azimuth angle of remote center point error.

Probe feed distance/mm	*x* direction				*y* direction				*x* and *y* directional random error relative parameter
	*μ* (mm)	*ε*_0_ (%)	RSD (%)	Confidence interval	*μ* (mm)	*ε*_0_ (%)	RSD (%)	Confidence interval	
0	8.30	7.78	14.40	(7.15, 9.44)	13.26	10.50	7.50	[12.30, 14.21]	0.342
30	8.40	6.67	12.80	(7.36, 9.43)	11.86	1.16	14.41	(11.22, 13.49)	0.758
60	9.54	6.00	12.50	(8.38, 10.69)	12.30	2.50	10.50	(11.05, 13.54)	0.840

**Table 4:** Analysis result of pitching angle of remote center point error.

Probe feed distance/mm	*x* direction				*z* direction				*x* and *z* directional random error relative parameter
	*μ* (mm)	*ε*_0_ (%)	RSD (%)	Confidence interval	*μ* (mm)	*ε*_0_ (%)	RSD (%)	Confidence interval	
0	8.72	14.73	12.97	(7.56, 9.95)	9.58	8.76	11.69	(8.50, 10.65)	0.741
30	7.46	1.84	14.98	(6.45, 8.46)	10.20	2.85	11.56	(9.16, 11.23)	-0.873
60	7.30	3.94	7.80	(6.75, 8.84)	8.90	15.23	9.10	(8.12, 10.67)	0.108

## Data Availability

The data used to support the findings of this study are available from the corresponding author upon request.
